The article "Data Analysis of Nursing Effects in Pediatric Gastroenterology Department under High Content Image Analysis Technology" was retracted in 2023. Reasons: signs of a paper mill; suspected computer-generated content; unreliable results or conclusions; lack of ethics approval or compliance.

# Data Analysis of Nursing Effects in Pediatric Gastroenterology Department under High Content Image Analysis Technology

**DOI:** 10.1155/2022/4302331

**Published:** 2022-07-30

**Authors:** Yanli Ma, Huini Liang, Yingying Jin

**Affiliations:** ^1^Department of Pediatric Digestive Infection, Gansu Provincial Maternity and Child-Care Hospital, Lanzhou 730050, Gansu, China; ^2^Department of Obstetrics and Gynecology, Gansu Provincial Maternity and Child-Care Hospital, Lanzhou 730050, Gansu, China; ^3^Department of Pediatric Respiratory, Gansu Provincial Maternity and Child-Care Hospital, Lanzhou 730050, Gansu, China

## Abstract

**Objective:**

Based on the nursing analysis of children aged 0∼3 in the Department of Gastroenterology, from the perspective of nursing methods and nutrition, bird's nest nursing and high-quality nursing methods were used to intervene children to help them improve their gastrointestinal conditions and sleep quality (Su-Jin, 2021).

**Methods:**

A total of 2465 healthy children under 3 years were selected, with normal action and intelligence and accompanied by their parents. Among them, there were 635 children in the observation group (O group) and 355 children in the reference group (R group) in the bird's nest nursing group, 572 children in the O group and 603 children in the R group in the other high-quality nursing group. The observation group received routine nursing, while the control group received nest nursing and quality nursing. The height growth rate, weight growth rate, brain weight growth rate, blood cell routine, and serum biochemical examination results of infants aged 6 months and 3 years in the O group, image analysis technology is used to analyze and discuss the gastrointestinal imaging examination of children, so as to conduct more detailed and accurate research.

**Results:**

Through the analysis and comparison of the physiological index data of 6-month-old and 3-year-old infants in the observation group and the reference group, and the satisfaction of parents, it was found that the children's physiological indexes, gastrointestinal digestion, weight gain, and brain weight gain rate through bird's nest care and high-quality care were slightly better than those in the observation group, and the parents' satisfaction was also slightly higher.

**Conclusion:**

Wei et al. (2020). By creating a comfortable environment and simulating the children's growth environment under the mother's care, it is found that the bird's nest care and high-quality care programs can calm children's emotions, increase children's appetite and digestion, so as to promote children's gastrointestinal digestion and achieve the goal of healthy growth (Wei et al, 2020). Finally, the conclusion is drawn that starting from the needs of children, scientific and correct gastrointestinal care and dietary nutrition should be used to promote the healthy growth of children.

The article "Data Analysis of Nursing Effects in Pediatric Gastroenterology Department under High Content Image Analysis Technology" was retracted in 2023. Reasons: signs of a paper mill; suspected computer-generated content; unreliable results or conclusions; lack of ethics approval or compliance.

## 1. Introduction

Infants, that is, children born to the age of three, different nutrition is required at different growth and development stages, and before the age of three is the first period of rapid growth and development of infants. During this period, children's physiological indicators and immune functions are relatively fragile and vulnerable to external influence and invasion due to different physiological structure characteristics and immune system perfection. Therefore, the nutrition supply in their growth stage needs to be particularly cautious and important. Because parents do not pay enough attention to nutrition knowledge, and influenced by traditional ideas, their understanding of nutrition still stays in the accumulation of quantity, they often ignore the types, structures, and combinations of nutrients. Reasonable nutrition supply plays a decisive role in their physical development, functional development, and immune function, and even affects their eating habits and healthy growth.

Physiological hunger is human's instinct. The food that the human body can extract, digest, absorb, and use can provide nutrients for human growth while meeting human physiological needs. Foods that people can mobilize include protein, fat, carbohydrates, water, and other minerals to provide energy and regulate physiological functions for the human body.

When children have digestive problems, they should seek medical attention in time. Medical image analysis refers to the combination of comprehensive medical images, digital image processing and analysis, artificial intelligence, and other technologies. The traditional medical image diagnosis of gastroenterology has great limitations. Using high content image analysis technology to diagnose children's digestive diseases will be more intuitive and accurate.

In view of the special digestive tract and picky food intake of infants and young children, we should take reasonable nursing and nutritional intervention and feed them scientifically and actively to ensure their physical and mental health. In this paper, bird's nest nursing and high-quality nursing are used to intervene them, and scientific nursing methods are used to serve them, comfort their emotions, and help them stabilize their character, so as to make them sleep quickly and help them eat and digest. Image analysis technology was used to track and analyze the gastrointestinal performance and physiological indicators of children regularly, and their nursing situation was evaluated.

The article "Data Analysis of Nursing Effects in Pediatric Gastroenterology Department under High Content Image Analysis Technology" was retracted in 2023. Reasons: signs of a paper mill; suspected computer-generated content; unreliable results or conclusions; lack of ethics approval or compliance.

## 2. Literature Resource

Among them: in the relevant literature of the bird's nest nursing group:

Literature [1] 133 cases in the observation group(O group) and 133 cases in the reference group (R group) [1]. Literature [2] 125 cases in the O group and 132 cases in the R group [2]. Literature [3] 140 cases in the O group and 140 cases in the R group [3]. Literature [4] 130 cases in the O group and 130 cases in the R group [4]. Literature [5] 107 cases in the O group and 120 cases in the R group [5];

In the literature related to the quality care group:

Literature [6] 95 cases in the O group and 95 cases in the R group [6]. Literature [7] 86 cases in the O group and 95 cases in the R group [7]. Literature [8] 105 cases in the O group and 105 cases in the R group [8]. Literature [9] 110 cases in the O group and 110 cases in the R group [9]. Literature [10] 63 cases in the O group and 60 cases in the R group [10]. Literature [11] 113 cases in the O group and 138 cases in the R group [11].

## 3. Statistical Methods

### 3.1. Nursing Path

#### 3.1.1. Experimental Group

Give the bird's nest nursing. Since the newborn children are soft and have strong dependence on the mother, the nursing staff will use the warm and comfortable bird's nest suitable for the body radian of infants and young children as the bed for infants and young children to rest, so as to increase the comfort of children's sleep. Adjust the softness and hardness of the bed and the light intensity according to the age of the child, disinfect the wet diapers, close fitting clothes and toiletries regularly, keep the children clean and give nutritional feeding regularly, and ensure reasonable exercise and nutritional absorption.

The high-quality nursing service mainly carries out nursing through hospitalization, intervenes with professional means, gets up every morning, cleans and soothes them, and gives them scientific nutritious meals. Observing the absorption of urine and feces is helpful to find problems in the nursing process. Moreover, a reasonable sleeping position can improve the sleep quality of infants and help them digest and stabilize their emotions. The overall comfortable environment can also make children relax and play a positive role in growth and digestion.

#### 3.1.2. Reference Group

In the nursing of the experimental group, the control group adopted the routine nursing mode, regularly changing and washing clothes, feeding food according to their preferences, monitoring routine physiological indicators, and carrying out other aspects of nursing according to the actual situation of children.

### 3.2. Patient Screening and Grouping Methods

In this study, 2465 normal and healthy children aged 0 to 3 years were selected, with normal development, no intestinal dysfunction, functional disorders caused by other drugs, and organic functional diseases. Normal action and intelligence, accompanied by parents. There were 635 children in the O group and 355 children in the R group in the bird's nest nursing group, 572 children in the O group and 603 children in the R group in the other high-quality nursing group. Through the analysis and comparison of various physiological index data of infants in the O group and the R group, it has a significant statistical significance.

The article "Data Analysis of Nursing Effects in Pediatric Gastroenterology Department under High Content Image Analysis Technology" was retracted in 2023. Reasons: signs of a paper mill; suspected computer-generated content; unreliable results or conclusions; lack of ethics approval or compliance.

In this study, both the *T* and *P* values of the bivariate *t* tests were obtained from the bivariate *t*-test procedure, in which *t* value is the value of the output result. *P* value is the log value of the output result. Subject to the length, calculation algorithm for the *T* value (value) The formula is as (1):

(1) $$\begin{array}{c} t_{\text{Value}}=\frac{\bar{x}-\mu }{\sigma_{x}\sqrt{n-1}},\bar{x},\\ \mu =\frac{1}{n,m}\sum_{i=1}^{n,m}x_{i},\\ \sigma_{x}=\frac{1}{n-1}\sqrt{\sum_{i=1}^{n}{\left(x_{i}-\bar{x}\right)}^{2}}. \end{array}$$

where $\bar{x}\;$ is the arithmetic mean of the investigated sample sequence, *μ*  is the average value of the reference sample sequence, n is the number of nodes of the investigated sample sequence, *m* is the number of nodes in the reference sample sequence, and *σ*_*x*_  is the standard deviation rate of the investigated sample sequence.

### 3.3. Observation Contents and Tracking Test Items

General surgical examination: the growth rate of height, weight and brain weight are the physiological indicators of children's physical examination. Through these indicators, the growth and development of children can be measured, and the growth and development of children can be detected by comparison.

Routine examination of blood cells: white blood cells, red blood cells, and platelets (the proportion of patients with statistical abnormalities, high/low) are indicators for blood item evaluation. They are tested to evaluate whether the blood routine meets the standard. Children with low red blood cells have the tendency of anemia, and high white blood cells indicate the existence of inflammation in their bodies, These indicators can be used to evaluate children's physical health and nutrition tracking.

Serum biochemical examination: the indicators of protein, iron, and trace elements are the monitoring of trace elements in children, and the nutritional absorption of children is tracked according to the data of these trace elements. The imbalance of trace elements can lead to abnormal growth. Most children with anorexia will have zinc deficiency in the detection, while the proportion of iron deficiency anemia in children is not small. The detection of trace elements can balance the nutritional collocation.

The article "Data Analysis of Nursing Effects in Pediatric Gastroenterology Department under High Content Image Analysis Technology" was retracted in 2023. Reasons: signs of a paper mill; suspected computer-generated content; unreliable results or conclusions; lack of ethics approval or compliance.

Medical imaging examination: endoscopic ultrasonography, electronic esophagogastroscopy, colonoscopy, CT, magnetic resonance imaging, etc., are used to perform gastrointestinal reconstruction angiography to determine whether there are organic lesions in the gastrointestinal tract.

## 4. Comparison of Nutritional Data of 6-Month-Old Newborns

According to different nursing methods for newborns, the newborns were examined by general surgery, medical imaging, blood cell routine, and serum biochemistry every month. We record and count the data of all inspection results. Image analysis technology was used to analyze the influence of examination results to adjust different nursing methods. The height, weight, brain weight, blood cell routine, and serum biochemical changes of the two groups of newborns after 6 months were compared. The specific data are as follows: Table 1.

From Table 1, it can be found that the data of height growth, weight growth, and brain weight growth of general nursing path, bird's nest nursing and high-quality nursing are statistically significant (*P* < 0.05), while the data of observation indexes of bird's nest nursing and high-quality nursing are not statistically significant (*P* > 0.05). According to the data in Table 1, as shown in Figure 1 below, the differences of the three groups of data can be more clearly compared visually;

As can be seen from Figure 1, the height, weight, and brain development of bird's nest nursing and high-quality nursing methods are better than those of general path nursing methods. However, in terms of weight and brain development, quality care is better. However, bird's nest nursing and high-quality nursing have their own advantages for the development of newborns, and their advantages and disadvantages are still unclear.

Table 1 shows the general surgical examination items for newborns. The following table is the statistical data of abnormal blood cell routine and serum life examination results of newborns at the age of 6 months. The detailed data are shown in Table 2.

As can be seen from Table 2, there were significant differences in the results of routine blood cell and serum biochemical tests between routine nursing, bird's nest nursing and high-quality nursing, and the results were statistically significant (*P* < 0.05), while there was no significant difference between bird's nest nursing and high-quality nursing, and there was no significant difference in infant growth and biochemical indicators. We make the following histogram 2 according to the data in Table 2.

The article "Data Analysis of Nursing Effects in Pediatric Gastroenterology Department under High Content Image Analysis Technology" was retracted in 2023. Reasons: signs of a paper mill; suspected computer-generated content; unreliable results or conclusions; lack of ethics approval or compliance.

It can be seen from Figure 2 that the contents of blood cells, blood protein, heme, and trace elements in 6-month-old newborns with high-quality care and bird's nest care are lower than those under the general path of care, while the abnormal content level of high-quality care is the same as that of bird's nest care.

## 5. Comparison of Nutritional Data of 4 Newborns Aged 3 Years

The newborns who adopt general nursing path, high-quality nursing method and bird's nest nursing method are tracked and investigated from birth until they reach the age of three. The height, weight, and brain development data of these newborns are recorded annually. These statistical data are statistically analyzed to obtain Table 3:

Rule regularities from Table 3, weight and brain weight is the same as that of 6-month-old newborns. The height, weight, and brain weight of newborns growing up under general path nursing are lower than those growing up under bird's nest nursing and high-quality nursing. The difference is that the growth rate of height, weight, and brain weight of high-quality nursing children at the age of 3 weeks is higher than that of bird's nest nursing, Although the data gap is not particularly obvious, we make Figure 3 according to the data in Table 3.

It can be seen from Figure 3 that the weight, height, and brain weight of children who grow up through high-quality nursing are the best. Although the observation indexes of children who grow up under bird's nest nursing are slightly worse than those of high-quality nursing, they are much better than those of children who grow up under general nursing. This also shows that using good nursing methods to feed newborns will be beneficial to the development of newborns.

According to the follow-up records of three-week-old children who grew up under the general nursing mode, bird's nest nursing mode and high-quality nursing mode from birth, these children were subjected to routine blood cell and serum biochemical examination every year, and the data of these examination results were statistically analyzed to obtain the data in Table 4.

In Table 4, it can be seen from the data of blood cell routine and serum biochemical examination results that the law is similar to that of 6-month-old blood cell routine and serum biochemical examination results. The abnormal rate of blood cell routine and serum routine examination results of 3-week-old newborns with general nursing method is higher than that of newborns with bird's nest nursing and high-quality nursing, There was no significant difference in the abnormal rate of blood cell routine and serum biochemical examination results of bird's nest nursing. We make the following Figure 4 according to the data of blood cell routine and serum biochemical examination results in Table 4.

The article "Data Analysis of Nursing Effects in Pediatric Gastroenterology Department under High Content Image Analysis Technology" was retracted in 2023. Reasons: signs of a paper mill; suspected computer-generated content; unreliable results or conclusions; lack of ethics approval or compliance.

Figure 4 shows that the results of routine blood cell and serum biochemical examination of children with bird's nest care and high-quality care are better than those of general path care, which shows that scientific care for newborns at birth is conducive to the healthy growth of children.

## 6. Comparison of Satisfaction of Routine Nursing Families of Newborns

A questionnaire survey was conducted on newborns who adjusted different nursing methods after using high content image analysis technology, so that the families of these newborns can evaluate these nursing methods. The specific satisfaction evaluation table is shown in Table 5.

In Table 5, a total of 2465 newborns' families were surveyed by questionnaire. From the data of the satisfaction form, it was found that the number of completely dissatisfied with high-quality care accounted for only 6.3% of all newborns' families who received high-quality care, which showed that 93.7% of them agreed with high-quality care. The number of people who agree with the bird's nest nursing method is less than that of high-quality nursing, but it is also much higher than that of general path nursing. According to the data of the above satisfaction statistical table, see Figure 5.

It is shown in Figure 5 that the number of people who are satisfied with high-quality care accounts for the most, the number of people who are dissatisfied accounts for the least, the number of people who are satisfied with bird's nest care accounts for the medium, the number of people who are satisfied with general care accounts for the least, and the number of people who are dissatisfied accounts for the most.

## 7. Critical Mate Discussion on Nursing in Pediatric Gastroenterology Department

With the development of society, people's living standards have gradually improved, especially after the change of population structure, the child birth rate has decreased, and people pay more and more attention to children's health. Now, with the improvement of living standards, some obese children have increased significantly, but their weight is not equal to health. Therefore, children's physical and mental health care has become the focus of attention.

Children aged 0 to 3 are vulnerable to external influence and have low immunity since they leave the mother. Intestinal digestion is fragile, which will bring certain risks to their health. Therefore, certain nursing measures are needed to intervene to help them grow healthily. Xiaohua said in the study that endoscopy can get a more accurate and comprehensive judgment of the patient's condition, which can also better monitor the intestinal changes of children. [12] Using image analysis technology to analyze and process images can assist doctors in qualitative or quantitative analysis of the diseased parts and greatly improve the reliability of medical diagnosis. Infants of six months age are mostly breastfed, and their mother's eating habits have a great impact on their intestinal digestion. Their nursing usually adopts bird's nest nursing and high-quality nursing scheme. By simulating the maternal environment, they can calm their emotions, provide a comfortable environment, increase their sleep quality, and help to improve their hair growth and development level.

The article "Data Analysis of Nursing Effects in Pediatric Gastroenterology Department under High Content Image Analysis Technology" was retracted in 2023. Reasons: signs of a paper mill; suspected computer-generated content; unreliable results or conclusions; lack of ethics approval or compliance.

After six months, the growth and development of infants' bodies began to accelerate, and their appetite began to increase slowly, so they needed more nutritional supplies. At this time, the role of breast milk began to weaken gradually and could not meet the needs of infants. Generally speaking, parents will supplement them with more nutritious food. Therefore, the combination of reasonable nutrition and nursing methods can promote children's thinking and cognitive ability and physical growth and development [13].

Before, the age of three is the first peak stage of children's development. At this time, children's body and psychology have a process of sudden learning and rapid progress. At this time, it not only needs a lot of nutritional supplies but also is extremely important for their psychological development. At this time, bird's nest nursing and high-quality nursing can calm their emotions and contribute to their sleep quality and physical development. Integrating nutritional care into child care can improve their physical and mental health and nutrition status [14].

## 8. Conclusion

Due to the diversification of diet, more and more people choose food, which leads to a serious shortage of fat and protein intake. Most people are more or less lack of trace elements. Eating habits have a certain impact on the body constitution, and the lack of variety will affect the absorption of some foods.

The study observed 2465 children. Different nursing methods were used by using high content medical image analysis technology to identify different lesions. The bird's nest nursing and high-quality nursing scheme can help children grow healthily by creating a comfortable environment and simulating the maternal growth environment, so as to calm children's emotions, increase children's appetite and digestion, improve their sleep quality, height speed, weight growth, and brain volume development. Through the comparison of the observation group, it is concluded that the physiological indexes of children with bird's nest nursing and high-quality nursing are slightly better than those in the observation group, and the satisfaction of parents is slightly higher.

The article "Data Analysis of Nursing Effects in Pediatric Gastroenterology Department under High Content Image Analysis Technology" was retracted in 2023. Reasons: signs of a paper mill; suspected computer-generated content; unreliable results or conclusions; lack of ethics approval or compliance.

According to the actual needs of children in the process of growth, correct scientific nursing methods and reasonable nutritional diet can promote children's gastrointestinal digestion, so as to further achieve the purpose of children's physical health and growth model. Using high content medical image analysis technology can efficiently and accurately process massive image information, eliminate human subjective factors, and improve the efficiency and accuracy of diagnosis. However, at present, the research in this field is not perfect, and there is still room for further exploration, which needs further development by scientists.

## Figures and Tables

**Figure 1:** Comparison of height growth, weight growth, and brain weight growth of newborns at 6 months of age in different nursing paths.

**Figure 2:** Comparison of blood cell and serum routine examination data of six-month-old newborns under different nursing methods.

**Figure 3:** Comparison of growth rate of height, weight, and brain weight at the age of 3 weeks under different nursing methods.

**Figure 4:** Comparison of blood cell and serum biochemical test data of 3-week-old children with different nursing methods.

**Figure 5:** Comparison of family satisfaction of newborns under different nursing methods.

**Table 1:** Comparison of height growth rate, weight growth rate, and brain weight growth rate of 6-month-old newborns (monthly average) (the data in the table are from relevant literature).

Grouping		Height growth	Weight growth	Brain weight growth
Group O	General path	4.05 ± 0.83	3.12 ± 0.46	10.60 ± 1.42
Group A	Bird's nest nursing	4.75 ± 0.91	3.38 ± 0.57	11.58 ± 1.92
Group B	Quality care	4.52 ± 0.95	3.42 ± 0.55	11.70 ± 1.87
*t *_OA_		3.695	5.418	8.367
*t *_OB_		3.702	5.134	8.759
*t *_AB_		28.355	35.742	19.257

**Table 2:** Blood cell routine and serum biochemical examination results of 6-month-old newborns (statistical abnormality rate) (the data in the table are from relevant literature).

Grouping		Blood corpuscle	Blood protein	Heme	Trace element
Group O	General path	1.25 ± 0.29	2.49 ± 0.25	6.91 ± 0.79	15.74 ± 2.15
Group A	Bird's nest nursing	0.75 ± 0.06	1.05 ± 0.13	3.27 ± 0.34	11.65 ± 1.83
Group B	Quality care	0.78 ± 0.08	1.09 ± 0.11	3.14 ± 0.32	11.49 ± 1.75
*t *_OA_		2.695	1.294	1.027	8.572
*t *_OB_		2.763	1.156	1.183	8.193
*t *_AB_		27.694	45.312	37.588	29.685

The article "Data Analysis of Nursing Effects in Pediatric Gastroenterology Department under High Content Image Analysis Technology" was retracted in 2023. Reasons: signs of a paper mill; suspected computer-generated content; unreliable results or conclusions; lack of ethics approval or compliance.

**Table 3:** Comparison of height growth rate, weight growth rate, and brain weight growth rate of newborns aged 3 weeks (average annual) (the data in the table are from relevant literature).

Grouping		Height growth	Weight growth	Brain weight growth
Group O	General path	10.22 ± 1.27	12.54 ± 1.49	89.65 ± 9.37
Group A	Bird's nest nursing	12.73 ± 1.68	14.62 ± 2.07	97.53 ± 10.52
Group B	Quality care	13.18 ± 1.73	14.76 ± 1.93	98.76 ± 9.89
*t *_OA_		4.297	5.925	6.571
*t *_OB_		4.682	5.473	6.823
*t *_AB_		27.365	42.376	39.657

**Table 4:** Results of routine blood cell and serum biochemical examination (statistical abnormality rate) (the data in the table are from relevant literature).

Grouping		Blood corpuscle	Blood protein	Heme	Trace element
Group O	General path	4.23 ± 0.48	5.38 ± 0.67	11.57 ± 1.52	17.68 ± 2.08
Group A	Bird's nest nursing	2.04 ± 0.25	2.76 ± 0.36	6.28 ± 0.76	11.29 ± 1.56
Group B	Quality care	1.96 ± 0.22	2.55 ± 0.33	6.94 ± 0.73	11.65 ± 1.73
*t *_OA_		2.695	1.294	1.027	8.572
*t *_OB_		2.763	1.156	1.183	8.193
*t *_AB_		27.694	45.312	37.588	29.685

**Table 5:** Comparison results of satisfaction of routine nursing families of newborns (the data in the table are from relevant literature).

Grouping		*N*	Satisfied	Basically satisfied	Dissatisfied	Completely dissatisfied
Group O	General path	1258	332 (26.4)	356 (28.3)	305 (24.2)	265 (21.1)
Group A	Bird's nest nursing	635	225 (35.4)	234 (36.9)	102 (16.1)	74 (11.7)
Group B	Quality care	572	217 (37.9)	223 (39.0)	96 (16.8)	36 (6.3)
*t *_OA_		—	2.685	3.650	1.415	2.083
*t *_OB_		—	2.245	3.187	1.658	1.594
*t *_AB_		—	24.693	35.734	19.274	5.392

## Data Availability

The data underlying the results presented in the study are available within the manuscript.
